This article has been retracted.

# Circular RNA circFAT1(e2) Promotes Colorectal Cancer Tumorigenesis via the miR-30e-5p/ITGA6 Axis

**DOI:** 10.1155/2021/9980459

**Published:** 2021-06-26

**Authors:** Fei Pan, Dongqing Zhang, Na Li, Mei Liu

**Affiliations:** Department of General Practice, Minhang Hospital, Fudan University, 170 Xinsong Road, 201199 Shanghai, China

## Abstract

circRNAs (circular RNAs) are a family of noncoding RNAs and have diverse physiological and pathological functions. However, the functions and mechanisms of circRNAs in the development and progression of colorectal cancer (CRC) remain largely unknown. Here, we aimed to explore the functions and roles of circFAT1(e2) in CRC. qRT-PCR revealed that circFAT1(e2) in CRC tumor tissues was upregulated compared with that in adjacent normal tissues and was also upregulated in CRC cell lines. Small interfering RNAs (siRNAs) against circFAT1(e2) were used to decrease the expression of circFAT1(e2) in HCT116 and RKO cells in vitro. The roles of circFAT1(e2) in CRC cell metastasis and proliferation were then determined by transwell and CCK-8 assays. The results showed that circFAT1(e2) silencing markedly suppressed CRC growth. Moreover, we identified circFAT1(e2) as a promoter of CRC metastasis. Knockdown of circFAT1(e2) evidently reduced HCT116 and RKO cell migration and invasion. Furthermore, the regulatory relationship between circFAT1(e2) and its target miRNAs was verified by a luciferase reporter assay. We demonstrated that circFAT1(e2) could sponge miR-30e-5p, which regulated the expression level of integrin *α*6 (ITGA6), the downstream target gene of miR-30e-5p. Rescue assays demonstrated that knockdown of miR-30e-5p enhanced CRC proliferation and migration via ITGA6. Taken together, our results reveal the novel oncogenic roles of circFAT1(e2) in CRC through the miR-30e-5p/ITGA6 axis.

## 1. Background

circRNA is a special type of noncoding RNA with a closed-loop structure in eukaryotic cells produced by the reverse splicing process. Due to the lack of a 5′-cap and poly-A tail, circRNAs are stable and difficult to digest by exonucleases [1, 2]. To date, little is known about circRNAs in human diseases due to the lack of powerful technical methods [3]. Recently, with the creation and improvements of next-generation sequencing technology and biological methods, emerging studies have demonstrated that circRNAs play important roles in human cancers [4–6]. In papillary thyroid carcinoma, overexpression of circRNA_102171 was found to promote cancer progression by activating the Wnt/*β*-catenin pathway in a CTNNBIP1-dependent manner [7]. CircKIAA1244, derived from gastric cancer tissue, is related to TNM staging and nodal metastasis and can be used as a new type of circulating biomarker for the detection of gastric cancer [8]. In cervical cancer, circRNA_0000285 can promote the proliferation and metastasis of cervical cancer by upregulating FUS and can be used as a potential target for cervical cancer treatment [9]. The effect of circRNAs on cancer has also become one of the hotspots of research [10]. Exploring the functions of circRNAs in cancers could provide novel biomarkers for cancer treatment [11, 12].

circFAT1(e2) originates from the second exon of FAT1 mRNA. According to a report by Fang et al. on gastric cancer, circFAT1(e2) can regulate the levels of the tumor suppressor gene RUNX1 (RUNX family transcription factor 1) in the cytoplasm by acting as a sponge for miR-548g and directly binding to YBX1 in the nucleus to inhibit protein function to suppress cancer progression [13]. However, circFAT1(e2) plays the opposite role in osteosarcoma. In osteosarcoma, circFAT1(e2) can adsorb miR-375 and reduce the inhibition of Yes-associated protein-1 expression by miR-375, thus promoting the growth and metastasis of tumor cells [14]. Thus, there is an urgent need to study the role of circFAT1(e2) in the dissemination and growth of colorectal cancer (CRC) cells.

To better understand the roles and mechanisms of circFAT1(e2) in CRC, researchers carried out several assays in the CRC cell lines HCT116 and RKO. Using the CCK-8 assay, it was found that the knockdown of circFAT1(e2) could significantly increase the proliferative ability of cancer cells. Transwell assays revealed that the metastatic ability of cancer cells significantly decreased after the knockdown of circFAT1(e2). Dual-luciferase reporter assays showed that circFAT1(e2) could act as a sponge to adsorb miR-30e-5p. Our findings provide a new biomarker for the prognosis and treatment of CRC patients.

## 2. Materials and Methods

### 2.1. Bioinformatics Analysis

In order to reveal the function of genes, we used the Database for Annotation, Visualization and Integrated Discovery (DAVID 6.8, https://david.abcc.ncifcrf.gov/) for GO annotation. We mainly analyzed biological processes (BP) and molecular functions (MF). *p* < 0.05 is considered statistically significant.

The potential targets of circFAT1(e2) were identified using circBank (http://www.circbank.cn/) and starBaseV2.0 (https://bigd.big.ac.cn/databasecommons/database/id/169) and the potential targets of miR-30e-5p were identified using TargetScan 7.2 (http://www.targetscan.org/vert_72/).

### 2.2. Experimental Samples

CRC samples were obtained at Minhang Hospital between July 2016 and March 2018. Ten paired CRC samples and normal tissues were used to detect circFAT1(e2) expression with real-time PCR. All experiments were approved by the Ethics Committee of Minhang Hospital of Fudan University. All the experimental samples of patients with CRC provided informed and written consent from themselves or their families.

### 2.3. Cell Lines and Cell Culture Experiments *In Vitro*

The human CRC cell lines HCT116 (CCL-247), Caco-2 (HTB-37), and RKO (CRL-2577) and one normal cell line FHC (CRL-1831) were purchased from ATCC (Manassas, Virginia, USA). All human CRC cell lines were cultured in Dulbecco's modified Eagle's medium (DMEM) (BI, Israel) with 10% foetal bovine serum (FBS) (BI, Israel) in a cell culture incubator containing 5% CO_2_ at 37°C.

### 2.4. RNA Extraction and qRT-PCR

Total RNA was extracted from CRC cells with TRIzol reagent (TaKaRa, Japan) following the instructions provided by the manufacturer. Reverse transcription and qRT-PCR were conducted with SYBR Premix Ex Taq (TaKaRa, Japan) in an Applied Biosystems 7900 HT Real-Time PCR System. GAPDH was used as the endogenous gene to calculate the relative gene expression. The relative expression was analyzed using the 2^−ΔΔ*CT*^ method.

### 2.5. Cell Transfection

Before transfection, CRC cells (2.5 × 10^4^/well) were cultured in a six-well plate for 24 hours. The siRNA was provided by GenePharma Co. Ltd. (Shanghai, China). The siRNA sequences were as follows: si-circFAT1 (e2) 5′-GAGACAGATTCCCGACAGTTAdTdT-3′, si-ITGA6 5′-CCTAGTGGGATATGCCTCCAGGTTA-3′, and si-NC 5′-UUCUCCGAACGUGUCACGUTT-3′. siRNA was transfected into CRC cells using Lipofectamine 2000 according to the manufacturer's instructions. Transfect all sequences into CRC cells for 48 hours to upregulate or downregulate the expression of circFAT1(e2) or ITGA6 in CRC cells.

### 2.6. Cell Growth Assay

A Cell Counting Kit-8 (CCK-8, Dojindo, Kumamoto, Japan) was used to detect cell proliferation capacity. A total of 2000 CRC cells after transfection in a 100 *μ*L medium were seeded in a 96-well plate (Corning, New York, USA). We supplemented 10 *μ*L of CCK-8 solution at 0, 24, 48, 72, and 96 hours and measured the optical density (OD) at 450 nm with a microtiter. The cell survival rate was expressed by absorbance. A total of 6 replicates were calculated under the same conditions to represent the results.

### 2.7. Transwell Assay

To determine the cell metastatic capacity, RKO and HCT116 cells in DMEM with 10% FBS were seeded in 24-well transwell chambers with (for cell invasion detection) or without (for cell migration detection) precoated Matrigel. Cells migrated through a polycarbonate membrane with 8 gas phase pores. The cell suspension was added to the upper chamber of the transwell (8 *μ*m pore size, Corning, NY, USA), and 100000 cells were tested for matrix gel invasion. After a 24-hour incubation, the filter membrane was removed from the chamber and washed three times with PBS and the medium and matrix were removed. Forty-eight hours later, the filter membrane was removed from the chamber and washed three times with PBS. The migrated/invaded cells were fixed with cold methanol for 10 minutes, stained with DAPI (10 *μ*g/mL) for 10 minutes, counted under a microscope, and photographed following the manufacturer's instructions.

### 2.8. Luciferase Reporter Assay

The plasmid (pGL3) containing wild-type or mutant circFAT1(e2) and ITGA6 3′-UTR targeted by miR-30e-5p was cloned into the pGL3 luciferase vector (Sangon Biotech (Shanghai) Co. Ltd.). Then, a Renilla luciferase vector was cotransfected into HEK (human embryonic kidney) 293T (ATCC-CRL-11268) cells by using Lipofectamine 2000 (Invitrogen, Carlsbad, CA) as a negative control. 293T cells were cultured in DMEM with 10% FBS and then maintained in a humidified atmosphere with 5% CO_2_ at 37°C. The luciferase activity was detected after 24 hours according to a Dual-Luciferase Reporter Assay System (Promega, Madison, Wisconsin, USA).

### 2.9. Statistical Analysis

All data in this study were expressed as the means ± SDs. The analysis of experimental data was calculated with SPSS 19.0 statistical software (IBM Inc., USA). The differences between groups were calculated using Student's *t*-test or one-way analysis of variance (ANOVA). We considered *p* < 0.05 to be statistically significant. The post hoc test that we used for pairwise comparisons with one-way ANOVA was LSD (least significant difference).

## 3. Results

### 3.1. Bioinformatics Analysis of circRNA circFAT1(e2) in CRC

circFAT1(e2) has been reported to be related to tumor progression. However, its roles in CRC remain largely unclear. In the present study, we first explored its potential roles in CRC using bioinformatics analysis. The bioinformatics analyses revealed that circFAT1(e2) was involved in regulating 20 biological processes (Figure 1(a)). The molecular function analysis demonstrated that circFAT1(e2) was significantly related to the following 15 regulatory mechanisms of organic cyclic compound binding: heterocyclic compound binding, nucleotide binding, catalytic activity, acting on DNA, catalytic activity, adenyl nucleotide binding, ATP binding, nucleic acid binding, purine nucleotide binding, ribonucleotide binding, purine ribonucleoside triphosphate binding, carbohydrate derivative binding, RNA binding, small molecule binding, and purine ribonucleotide binding (Figure 1(b)). The results indicated that circFAT1(e2) might be involved in regulating the occurrence and development of CRC through these pathways.

### 3.2. The Expression Levels of circRNA circFAT1(e2) and circFAT1(e2) in CRC Tissues Promote CRC Cell Proliferation

We validated circFAT1(e2) expression using 10 pairs of CRC samples. As shown in Figure 2(a), the relative expression level of circFAT1(e2) in CRC increased by an average of 7.3-fold compared with that in adjacent normal tissues. Collectively, these data suggest that circFAT1(e2) might be related to the progression of CRC. By detecting the circFAT1(e2) level in CRC cells, we found that circFAT1(e2) in RKO and HCT116 cells was highly expressed compared to that in HT29 cells (Figure 2(b)). Then, loss-of-function assays were applied using siRNAs specifically targeting this circRNA. In this study, we designed and tested two siRNAs to knockdown circFAT1(e2). siRNA2 knockout efficiency was low (data were not shown). Therefore, we used siRNA1 to explore the potential function of circFAT1(e2) in CRC (Figure 2(c)). In addition, we also tested the knockout efficiency of si-ITGA6 (Figure 2(d)). CCK-8 assay results showed that circFAT1(e2) knockdown inhibited the proliferative capability of HCT116 and RKO cells (Figures 2(e) and 2(f)).

### 3.3. circFAT1(e2) Knockdown Suppresses CRC Migration and Invasion

Transwell assays for migration and invasion were performed using si-circFAT1(e2), and the results indicated that circFAT1(e2) silencing reduced the migration and invasion of CRC cells through the chamber membrane (Figures 3(a) and 3(c)). The number of migrated HCT116 and RKO cells in the circFAT1(e2) knockdown group decreased by approximately 75% and 60%, respectively, compared to that in the control group (Figure 3(b)). The number of invaded HCT116 and RKO cells in the circFAT1(e2) knockdown group decreased by approximately 55% and 85%, respectively, compared to that in the control group (Figure 3(d)). These results demonstrate that silencing circFAT1(e2) inhibited the migration and invasion of CRC cells in vitro.

### 3.4. miR-30e-5p Is a Direct Target of circFAT1(e2)

Consequently, we identified potential miRNAs targeting circFAT1(e2). Numerous online database analyses indicated that miR-30e-5p might be a direct binding site of this circRNA (Figure 4(a)). The results demonstrated that there was a series of complementary binding sites between miR-30e-5p and circFAT1(e2). Moreover, dual-luciferase reporter assays showed that circFAT1(e2) could interact with miR-30e-5p (Figure 4(b)). Furthermore, the relative expression level of miR-30e-5p was increased in CRC cells after transfection with si-circFAT1(e2) (Figure 4(c)). However, the high expression of miR-30e-5p did not change the relative abundance of circFAT1(e2) (Figure 4(d)).  Figure 4(e) showed that miR-30e-5p and miR-30e-5p-in have higher overexpression and inhibition efficiency, respectively. Our results revealed that circFAT1(e2) acted as a miR-30e-5p sponge. The CCK-8 assay revealed that the high expression of miR-30e-5p very clearly inhibited the proliferation of CRC cells but the silencing of miR-30e-5p promoted this proliferation (Figures 4(f) and 4(g)). Furthermore, transwell assays demonstrated that miR-30e-5p overexpression appreciably reduced the metastatic ability of CRC cells (Figures 4(h)–4(k)).

### 3.5. ITGA6 Acts as the Functional Target of miR-30e-5p in CRC

Next, we explored the potential effect and possible targets of miR-30e-5p in CRC. The target mRNAs of miR-30e-5p were obtained with the TargetScan databases (Figure 5(a)). The results from a dual-luciferase assay confirmed that the relative fluorescence activity was obviously reduced after WT 3′-UTR ITGA6 was cotransfected with miR-30e-5p, indicating the interaction between miR-30e-5p and ITGA6 (Figure 5(b)). Moreover, upregulation or downregulation of miR-30e-5p decreased or enhanced ITGA6 expression (Figure 5(c)). Then, we conducted rescue assays to validate that miR-30e-5p suppressed CRC progression via ITGA6 (Figure 5(d)). Transwell and CCK-8 assays showed that the knockdown of ITGA6 reversed the effects of the miR-30e-5p inhibitor on cell migration and proliferation of RKO cells (Figures 5(e) and 5(f)). Therefore, we confirmed that ITGA6 was a possible target of miR-30e-5p in the development of CRC.

## 4. Discussion

It is well known that the overall survival rate of CRC patients after surgery remains low worldwide [15–17]. According to statistics in 2018, the number of new CRC cases ranks third and the mortality rate of this cancer ranks second among all cancers [18, 19]. Therefore, the identification of novel biomarkers is particularly important for the early diagnosis and monitoring of CRC. A considerable number of miRNAs are considered detection markers for CRC [20, 21]. For example, miR-21 and miR-92a can be detected in the serum samples of CRC patients and can be potential diagnostic markers. The high expression of serum miR-92a is related to the poor prognosis of patients with CRC [22]. miR-135b can be used as a molecular marker for early screening for CRC [1]. miR-106a is more stable than miR-135b, which can increase the sensitivity of faecal detection [23]. By microarray analysis, it was discovered that as many as 20 miRNAs were differentially expressed in CRC cells and the expression levels of these miRNAs increased or decreased in different cancer stages [24, 25]. The therapeutic markers of CRC are related to the use of clinical drugs. For example, clinical studies of patients treated with cetuximab showed that miR-31-5p was closely related to the stage of cancer development [26, 27]. miR-200C can be used as a molecular marker to monitor the progression of the disease, and its expression level in the sera of patients with stage IV CRC is markedly higher than that in the sera of early- and middle-stage patients [28, 29]. Similarly, studies have found that patients with relatively high expression levels of miR-224 have a poor prognosis [30].

circRNAs generally originate from the reverse splicing of linear RNA sequences and have various miRNA binding sites, thus acting as ceRNAs (competing endogenous RNAs) to affect their activity and inhibit the downregulation of downstream gene expression by miRNAs [31]. ceRNA is a transcript that can be mutually regulated at the posttranscriptional level by competing with shared miRNAs [32].The ceRNA network connects the function of protein-coding mRNA with the function of noncoding RNA (such as microRNA, long noncoding RNA, pseudogene RNA, and circular RNA) [33]. RNA transcripts act as ceRNAs or natural microRNA sponges; they communicate with each other and regulate expression by competing for binding to shared microRNAs [34]. ciRS-7 is the first circRNA that has been proposed to regulate the expression of multiple genes, including miR-7. ciRS-7 can regulate the expression of oncogenes by sponging miR-7 [35]. In placental mammals, miR-7 is tightly coupled with ciRS-7. At present, some evidence shows that miR-7 is related to a variety of pathways and diseases: as a direct regulator of *α*-synuclein, it plays a role in Parkinson's disease, it regulates the mTOR signaling pathway in pancreatic B cells to promote cell proliferation, and it directly targets and downregulates the central carcinogen in tumor-related signaling pathways, which has a significant tumor suppressor effect [36]. A large number of studies have confirmed that circRNAs play an essential role in regulating the occurrence and progression of cancer [37, 38], including circFAT1(e2) [13]. For instance, in osteosarcoma, circFAT1(e2) can sponge miR-375 to stimulate cancer cell growth and metastasis [14]. In gastric cancer, circFAT1(e2) can adsorb miR-548g to suppress the growth of cancer cells. These results show the complex roles of circFAT1(e2) as a regulatory factor in cancers [13]. Our results show that circFAT1(e2) can act as a ceRNA to competitively bind to downstream miR-30e-5p and reduce the abundance of miR-30e-5p in cells. Moreover, overexpression and downregulation of miR-30e-5p suppresses and enhances the migration and growth abilities of CRC cells.

ITGA6-encoding proteins are related to cell adhesion. The available evidence shows that ITGA6 is associated with the development of cancer and is involved in regulating the metastatic and invasive ability of cancer cells [39]. As an example, Brooks et al. found that the high expression of ITGA6 could enhance the invasiveness of breast cancer cells and stimulate the activity of tumor-initiating cells at the stage of tumorigenesis [40]. According to a report by Yamakawa et al., ITGA6 has an important effect on the adhesion ability of EVI1^high^ leukaemia cells. High expression of ITGA6 can enhance the adhesion ability of tumor cells and lead to poor prognosis of EVI1^high^ leukaemia patients [39]. Our results show that miR-30e-5p can suppress cancer cell proliferation and migration by reducing the expression of ITGA6 in CRC.

This study has limitations. circFAT1(e2) overexpression experiments to confirm the tumor-inducing effects of circFAT1(e2) should be performed. In future research, we will use databases and collect more clinical samples to explore the correlation between circFAT1(e2) and clinical parameters (including the TNM stage, histologic differentiation age, and survival time). Then, we will also explore the role of ITGA6 in the proliferation, migration, and invasion of CRC. In addition, we will further explore the sponge effect of circFAT1(e2) on miR-30e-5p to further clarify the mechanism of circFAT1(e2) in colorectal cancer, such as RNA pull down and RIP.

Taken together, the current work demonstrates that circFAT1(e2) enhanced the expression level of ITGA6 by suppressing miR-30e-5p expression, which promoted the invasion, migration, and proliferation of CRC cells. In short, this research provides a new target for screening, diagnosing, treating, and monitoring CRC.

## Figures and Tables

**Figure 1:** Bioinformatics analysis of circRNA circFAT1(e2) in CRC. (a) The bioinformatics analysis revealed that circFAT1(e2) was involved in regulating multiple biological processes. (b) The molecular functions analysis of circFAT1(e2).

**Figure 2:** The expression level of circRNA circFAT1(e2) in CRC tissues and circFAT1(e2) promoted CRC cell proliferation in vitro. (a) CircFAT1(e2) expression levels in CRC tissues and adjacent nonneoplastic normal tissues. Error bars represent the mean ± SD of at least three independent experiments. ^∗∗∗^*p* < 0.001 vs. control group. (b) The relative circFAT1(e2) expression to normal colorectal cell in 3 CRC cell lines such as HCT116, CaCO2, and RKO. Error bars represent the mean ± SD of at least three independent experiments. ^∗^*p* < 0.05 and ^∗∗^*p* < 0.01 vs. the control group. (c) The relative circFAT1(e2) expression to negative control in HCT116 and RKO cells after knockdown of circFAT1(e2) by si-circFAT1(e2). Error bars represent the mean ± SD of at least three independent experiments. ^∗^*p* < 0.05 and ^∗∗^*p* < 0.01 vs. the control group. (d) The relative ITGA6 expression to negative control in HCT116 and RKO cells after knockdown of ITGA6 by si-ITGA6. Error bars represent the mean ± SD of at least three independent experiments. ^∗^*p* < 0.05 and ^∗∗^*p* < 0.01 vs. the control group. (e, f) CCK-8 assays in CRC cell lines transfected with si-NC or si-circFAT1(e2). Error bars represent the mean ± SD of at least three independent experiments. ^∗^*p* < 0.05 and ^∗∗^*p* < 0.01 vs. the control group.

**Figure 3:** The knockdown of circFAT1(e2) inhibited the migration and invasion abilities of the CRC cells. (a, b) Transwell cell migration assay in CRC cells transfected with si-NC or si-circFAT1(e2). Error bars represent the mean ± SD of at least three independent experiments. ^∗∗^*p* < 0.01 and ^∗∗∗^*p* < 0.001 vs. the control group. (c, d) Transwell cell invasion assay in HCT116 and RKO cells transfected with si-NC or si-circFAT1(e2). Error bars represent the mean ± SD of at least three independent experiments. ^∗∗^*p* < 0.01 and ^∗∗∗^*p* < 0.001 vs. the control group.

**Figure 4:** miR-30e-5p was a direct binding site of circFAT1(e2). (a, b) The dual-luciferase report assay in 293T cells transfected with luciferase report plasmids containing circFAT1(e2) (circFAT1(e2)3′UTR-WT or circFAT1(e2)3′UTR-mut) with mimic-NC, miR-30e-5p, or miR-30e-5p-in. Error bars represent the mean ± SD of at least three independent experiments. ^∗^*p* < 0.05 miR-30e-5p vs. mimic-NC. ^#^*p* < 0.05 miR-30e-5p-in vs. inhibit-NC. miR-30e-5p-in represents the miR-30e-5p inhibitor. (c) The qRT-PCR assays of the relative expression level of miR-30e-5p to mimic-NC in CRC cells transfected with si-circFAT1(e2) or si-NC. Error bars represent the mean ± SD of at least three independent experiments. ^∗∗^*p* < 0.01 vs. the control group. (d) The qRT-PCR assays of relative circFAT1(e2) expression to mimic-NC in CRC cells transfected with mimic-NC or miR-30e-5p. Error bars represent the mean ± SD of at least three independent experiments. (e) The miR-30e-5p expression levels as determined by qRT-PCR in CRC cells transfected with mimic-NC, miR-30e-5p, or miR-30e-5p-in. Error bars represent the mean ± SD of at least three independent experiments. ^∗∗∗^*p* < 0.001 miR-30e-5p vs. mimic-NC. ^#^*p* < 0.05 miR-30e-5p-in vs. inhibit-NC. miR-30e-5p-in represents the miR-30e-5p inhibitor. (f) G CCK-8 assay in CRC cells transfected with mimic-NC, miR-30e-5p, or miR-30e-5p-in. Error bars represent the mean ± SD of at least three independent experiments. ^∗^*p* < 0.05 and ^∗∗^*p* < 0.01 miR-30e-5p vs. mimic-NC. ^#^*p* < 0.05 and ^##^*p* < 0.01 miR-30e-5p-in vs. inhibit-NC. miR-30e-5p-in represents the miR-30e-5p inhibitor. (h, i) Transwell migration assay in HCT116 cells transfected with miR-30e-5p or mimic-NC by Lipofectamine 2000. Error bars represent the mean ± SD of at least three independent experiments. ^∗^*p* < 0.05 miR-30e-5p vs. mimic-NC. (j, k) Transwell invasion assay in RKO cells transfected with miR-30e-5p or mimic-NC by Lipofectamine 2000. Error bars represent the mean ± SD of at least three independent experiments. ^∗∗∗^*p* < 0.001 miR-30e-5p vs. mimic-NC.

**Figure 5:** ITGA6 acted as a potential downstream binding site of miR-30e-5p in the process of CRC. (a, b) Dual-luciferase assay in 293T cells transfected with luciferase report plasmids containing ITGA6 3′UTR (wild type or mutant) with mimic-NC, miR-30e-5p, or miR-30e-5p-in. Error bars represent the mean ± SD of at least three independent experiments. ^∗^*p* < 0.05 miR-30e-5p vs. mimic-NC. ^#^*p* < 0.05 miR-30e-5p-in vs. inhibit-NC. (c) Relative mRNA of ITGA6 in 293T cells which transfected with miR-30e-5p-in, miR-30e-5p, or mimic-NC. Error bars represent the mean ± SD of at least three independent experiments. ^∗^*p* < 0.05 miR-30e-5p vs. mimic-NC. ^#^*p* < 0.05 miR-30e-5p-in vs. inhibit-NC. (d) The expression levels of ITGA6 in 293T cells which transfected with si-ITGA6, miR-30e-5p-in, or mimic-NC. Error bars represent the mean ± SD of at least three independent experiments. ^∗^*p* < 0.05 si-ITGA6 vs. si-NC. ^#^*p* < 0.05 miR-30e-5p-in vs. inhibit-NC. (e) Cell migration assay and (f) CCK-8 assay in 293T cells which transfected with si-ITGA6, miR-30e-5p-in, or mimic-NC. Error bars represent the mean ± SD of at least three independent experiments. ^∗^*p* < 0.05 vs. the control group.

## Data Availability

The datasets used and/or analyzed during the current study are available from the corresponding author on reasonable request.
